# Huayu Sanjie Enema Liquid Relieves Pain in Endometriosis Model Rats by Inhibiting Inflammation, Peripheral Sensitization, and Pelvic Adhesion

**DOI:** 10.1155/2022/5256578

**Published:** 2022-06-28

**Authors:** Chunxiao Zong, Lu Sun, Xin Xu, Xiaoou Xue

**Affiliations:** ^1^Dongzhimen Hospital, Beijing University of Chinese Medicine, Beijing, China; ^2^Yuquan Hospital of Tsinghua University, Beijing, China

## Abstract

The objective of this study is to observe the effect of relieving pain of Huayu Sanjie enema liquid (HYSJ-EL) on endometriosis model rats and to explore its mechanism of action. Of 24 female Sprague Dawley rats, six were randomly selected as the sham operation group (normal control group). The remaining rats were used to establish rat models of endometriosis through autologous endometrial transplantation combined with estrogen injection. Successfully modeled rats were randomly divided into the model, indomethacin (Western medicine group), and HYSJ-EL (Chinese herbs group) treatment groups. The thermal pain threshold of rats was measured, and hematoxylin and eosin staining was used to observe pathological changes after sampling. Serum levels of prostaglandin E2 (PGE2), interleukin-6 (IL-6), macrophage inflammatory protein-2 (MIP-2), plasminogen activator inhibitor-1 (PAI-1), and transforming growth factor-*β* (TGF-*β*) were measured using an enzyme-linked immunosorbent assay (ELISA). Furthermore, the protein and mRNA expression levels of transient receptor potential vanilloid-1 (TRPV1) and tumor necrosis factor-*α* (TNF-*α*) in the endometrium and endometriotic lesions were measured using Western blotting and quantitative real-time PCR assays, respectively. Compared to the model group, the heat pain threshold of rats in the HYSJ-EL group was significantly increased (*P* < 0.01), and the serum levels of PGE2, IL-6, MIP-2, PAI-1, and TGF-*β* were significantly decreased (*P* < 0.01), as well as the expression of TRPV1 and TNF-*α* protein and mRNA in the tissue of the ectopic lesion was significantly decreased (*P* < 0.05). These results indicate that the Huayu Sanjie enema liquid exerts analgesic effects on endometriosis by inhibiting inflammation, peripheral nerve sensitization, and pelvic adhesion.

## 1. Introduction

Endometriosis (EMs) is a common gynecological disease with various clinical manifestations in which functional endometrial tissue grows outside the uterine cavity. Chronic pelvic pain is its main clinical symptom, which seriously affects the health and quality of life of patients [1]. Therefore, alleviating pelvic pain is one of the main objectives and evaluation indicators for the treatment of EMs [2, 3]. The underlying mechanisms responsible for the occurrence of pelvic pain in EMs have not yet been fully understood, and a detailed study of its internal pathogenesis will be beneficial in finding ideal treatments. Recent studies have shown that potential factors involved in the appearance of pelvic pain from EMs include inflammation, estrogen, nerve fibers, pelvic adhesion, central nerve sensitization, and peripheral nerve sensitization [4].

Pelvic pain from EMs is closely associated with local inflammation of the pelvis. EMs is an aseptic inflammatory disease. Many inflammatory factors are involved in the formation of EMs and mediate the production of pelvic pain [5]. Studies have shown that the concentration of inflammatory factors IL-6, TNF-*α*, PGE2, and MIP-2 in serum are correlated with the degree of pain from EMs [6–9].

Peripheral nerve sensitization plays an important role in the development of EMs pain. Inflammatory factors released from localized EMs lesions will activate and sensitize peripheral nerve fibers so that the relevant ion channels located on the end surface of pain receptors are activated or sensitized to excite nociceptors, thus generating action potentials and causing pain. The expression of TRPV1, a membrane ion channel receptor, has been shown to be positively correlated with the degree of chronic pelvic pain [10].

Pelvic adhesion is a cause of pain in patients with EMs. Scar contracture and adhesion-induced fibrosis lead to the formation of a band between tissues, which causes pain by pulling or twisting tissues and organs during exercise, standing, and defecation. The degree of pelvic adhesions in EMs patients is related to dysmenorrhea, chronic pelvic pain, and pain during intercourse [11]. Transforming growth factor-*β* (TGF-*β*) and plasminogen activator inhibitor-1 (PAI-1) can promote the formation of pelvic adhesions. Studies have shown that the levels of TGF-*β* and PAI-1 in the peritoneal fluid of EMs patients were significantly higher than those in individuals without EMs [12, 13].

Chinese herbs can improve the symptoms of EMs [14]. Traditional Chinese medicine (TCM) believes that blood stasis is the essential pathological basis of EMs. Promoting blood circulation to remove blood stasis is a common treatment. EMs lesions are mainly located in the pelvic cavity, rectum, and sigmoid colon and are also located in the pelvic cavity, adjacent to the uterus. A TCM enema can directly absorb, disperse, and infiltrate drugs into pelvic tissues through the intestinal mucosa and promote local blood circulation and metabolism of pelvic tissues. Compared with oral administration, the TCM retention enema avoids the first-pass effect of the liver [15]. The Huayu Sanjie Enema Liquid is a TCM enema formulation. It originates from Taohong Siwu Decoction (*Angelica sinensis, Rhizoma Chuanxiong, Radix Paeoniae Rubra, Radix Rehmanniae, Semen Persicae,* and *Flos Carthami*), a classic prescription for promoting blood circulation and removing blood stasis in the “Yizong Jinjian” proposed by Wu Qian, a physician in the Qing Dynasty. It has the effect of promoting blood circulation, removing blood stasis, and relieving pain. In addition, *Sparganii Rhizoma* and *Rhizoma Curcumae* in this prescription can break down blood and eliminate symptoms. *Turtlenail* and *Amydae carapax* can soften and evacuate the lump. *Radix Salviae Miltiorrhizae* can remove blood stasis. *Forsythiae and Flos Lonicerae* can remove heat and dissipate blood stasis. *Radix Achyranthis Bidentatae* and *Akebia stem* can dredge blood vessels and stimulate blood circulation. The whole prescription has the effects of promoting blood circulation to remove blood stasis, softening to dissipate blood stasis, clearing heat, and detoxicating [16]. Previous clinical studies have shown that the Huayu Sanjie Enema Liquid is effective for alleviating dysmenorrhea and chronic pelvic pain in patients with EMs. The purpose of this study is to observe the therapeutical effects of Huayu Sanjie enema liquid on EMs model rats and their influence on inflammation, peripheral nerve sensitization, and pelvic adhesion and to explore the mechanism of Huayu Sanjie Enema Liquid in the treatment of pelvic pain in EMs.

Indomethacin is a nonsteroidal anti-inflammatory drug with anti-inflammatory and analgesic effects, which can be used in the treatment of EMs pain in the clinic [17]. Therefore, we selected indomethacin as the positive control drug in our experiments. Indomethacin has a variety of dosage forms, including tablets, suppositories, and capsules. Although suppositories can be administered through the rectum, it is difficult to melt the suppositories but . the enema liquid of the experimental drug Huayu Sanjie is liquid. Thus, indomethacin capsules were selected as the dosage form to prepare the suspension, so that both the Chinese medicine administration group and the positive control group were used as a liquid formulation to avoid confounding effects.

## 2. Materials and Methods

### 2.1. Animals

A total of 24 SPF female Sprague Dawley rats, 8–10 weeks old, weighing 180–230 g, were purchased from Vital River Laboratory Animal Technology Co., Ltd. (Beijing, China). The animals were raised in a controlled environment animal room of Dongzhimen Hospital of Beijing University of Chinese Medicine at a room temperature of 24°C, humidity of 60%–70%, and an alternate photoperiod of 12 hours. The rats could freely eat and drink. Animal experiments strictly complied with the requirements of the Experimental Animal Welfare and Ethics Committee of Dongzhimen Hospital, Beijing University of Chinese Medicine (No. BUCMDZM-2020-16).

### 2.2. Chemicals and Reagents

Huayu Sanjie Enema Liquid was purchased from Qinghai Ruicheng Pharmaceutical Co., Ltd. (Shanghai, China). It consists of *Angelica sinensis, Rhizoma Chuanxiong, Radix Paeoniae Rubra, Radix Rehmanniae, Semen Persicae, Flos Carthami, Radix Achyranthis Bidentatae, Sparganii Rhizoma, Rhizoma Curcumae, Radix Salviae Miltiorrhizae, Turtlenail, Amydae carapax, Akebia stem, Forsythiae,* and *Flos Lonicerae.*

Indomethacin capsules were purchased from Hebei Yongfeng Pharmaceutical Co., Ltd. (Shijiazhuang, China). The dosage for Sprague Dawley (SD) rats was converted according to the equivalent dose coefficient conversion algorithm.

Rat PGE2, IL-6, TNF-*α*, MIP-2, PAI-1, and TGF-*β* ELISA kits were purchased from the Nanjing Jiancheng Institute of Bioengineering (Nanjing, China). Rabbit anti-TRPV1 antibody and rabbit anti-TNF-*α* antibody were purchased from Beijing Biosynthesis Biotechnology Co., Ltd. (Beijing, China). Protein extracts and protease inhibitors were purchased from Beijing Biosynthesis Biotechnology Co., Ltd. (Beijing, China). The SuperScript III Reverse Transcription kit and SYBR qPCR mix were purchased from Thermo Fisher Scientific Co., Ltd. (Shanghai, China).

### 2.3. Establishment of the Rat Model of Endometriosis

After adaptive feeding for 1 week, 6 rats among the 24 rats were randomly selected as the sham operation group (Normal control group). The remaining rats were used to establish rat models of EMs through autologous endometrial transplantation combined with injection of estrogen under sterile conditions [18]. After weighing, the rats were anesthetized by intraperitoneal injection of 2% pentobarbital sodium (30 mg/kg), fixed on the surgical plate, and prepared for abdominal skin and routine disinfection. The breakthrough point was selected at 1 cm above the urethral orifice, and a 1.5–2.0 cm incision was made along the front midline longitudinally. The abdominal wall was opened layer by layer and the rat “Y” type uterus was identified after entering the abdomen. The right uterus was separated and ligation of both ends was performed. An approximately 1 cm sample of the middle section of uterine tissue was quickly transferred into the dish and washed with saline. The tubular uterus was longitudinally cut with ophthalmic scissors and cut into fragments of approximately 5 mm × 5 mm in size. The endometrial surface of the uterus was sutured toward the peritoneum of the left peritoneal vascular rich area so that it was completely attached to the abdominal wall. After checking for no active bleeding, an intraperitoneal injection of penicillin was administered to prevent infection, and the abdomen was closed step by step, followed by disinfection of the incision. Penicillin was continuously injected intraperitoneally for three days after the operation to prevent infection. The sham operation group was prepared and anesthetized prior to the operation. The right uterus was located without any invasive surgery, and the left peritoneal region was sutured with 2 stitches of 5–0 nylon suture.

Starting on day 2 after the operation, 0.1 mg/kg estradiol benzoate was injected intramuscularly twice a week. The rats in the sham operation group were given the same amount of normal saline. After 4 weeks of modeling, an open view of the modeling outcome was performed to allow the naked eye to observe the increase in graft volume and the surface of the graft angiogenesis. The graft appeared as a small cystic nodule containing bright liquid, which confirmed the success of the EMs-rat model.

### 2.4. Animal Grouping and Treatments

The 24 rats were randomly divided into 4 groups with 6 rats in each group: sham operation group (Normal control group), model group, positive control group (indomethacin group), and Huayu Sanjie Enema Liquid group (HYSJ-EL group) [19]. After 4 weeks of modeling, each rat in the HYSJ-EL group was given a 2.5 mL enema of a drug solution equivalent to 5 mL/kg of Huayu Sanjie enema solution. Each rat in the positive control group was given a 2.5 mL enema of mixed suspension prepared with 2.5 mg/kg indomethacin; the sham operation group and the model group were given the same volume of normal saline enema, once per day, continuously for 4 weeks. The administration method was as follows: after the rats were fixed by a fixer, the disposable anal tube was inserted into the rectum of the rats at 5 cm, and a small amount of multiple administrations were conducted until all 2.5 mL of the liquid was imported.

### 2.5. Detection of Thermal Pain Threshold in Rats

The thermal pain threshold of the rats was measured using the light tail-flicking method after 4 weeks and 8 weeks of modeling. The lower 1/3 of the rat tail was taken as the light stimulation point, and the light power value of the YLS-12A rat tail light pain meter was set at 38 W. The incubation period from the beginning of irradiation to the tail flick reaction was measured twice continuously, and the interval time was 5 min. The mean value was taken as the pain threshold.

### 2.6. Sample Collection and Histological Observation

After 8 weeks of modeling (Day 2 after the last enema), the rats were anesthetized and serum, normal endometrium, and ectopic endometrium were collected. The size of ectopic lesions was measured and the lesion volume was calculated as follows: lesion volume = 1/2 × maximum transverse diameter × (vertical to the maximum transverse diameter)^2^. The ectopic endometrial tissue and normal endometrial tissue in the sham operation group were fixed with 4% paraformaldehyde, routine paraffin embedding, and 5 *μ*m continuous slices were prepared followed by hematoxylin and eosin (HE) staining, neutral tree film sealing, and the morphology of endometrial tissue was observed under an optical microscope. Masson staining was used to observe intimal fibrosis.

### 2.7. Enzyme-Linked Immunosorbent Assay

Rat serum was taken and the concentration of PGE2, IL-6, MIP-2, PAI-1, and TGF-*β* in serum was determined using ELISA according to the manufacturer's protocol. The optical density (OD) of each well was measured at 450 nm wavelength by an enzyme-labeled instrument. The standard curve was drawn according to the kit instructions, and the concentrations were calculated.

### 2.8. Western Blotting Analyses

Ectopic endometrial tissue or eutopic endometrial tissue in the sham operation group was cut on ice, added with cell lysate, and the tissue was homogenized in the ice bath. At 4°C, the supernatant was centrifuged at 12,000 rpm for 15 min and the buffer solution was added. The protein content was determined using the BCA protein concentration determination kit. The protein was normalized to 5 mg/mL and loaded onto SDS-PAGE gels for electrophoresis. After electrophoresis, the protein bands isolated from the gel were transferred to the PVDF membrane by transfer electrophoresis. The PVDF membrane was then immersed in the blocking solution and gently shaken for 1 h. The membrane was incubated at 4°C overnight with TRPV1, TNF-*α*, and *β*-actin primary antibodies (dilution ratio 1 : 1000). After being washed with TBST, the membrane was incubated at 37°C for 1 h with a horseradish peroxidase-labeled secondary antibody. After being washed with TBST, the ECL reagent was evenly spread on the surface of the PVDF membrane and allowed to react at room temperature for 4 min. The liquid on the membrane was shaken off and placed in the chemiluminescence imaging system to analyze the optical density value of the strip. The relative expression of the target protein was calculated as the gray value of the target protein/the gray value of the internal reference *β*-actin.

### 2.9. Quantification of mRNA by RT-PCR

Total RNA was extracted using the TRIZOL reagent and reverse transcribed into cDNA using the Reverse Transcription Kit Superscript III. The mRNA level was detected by quantitative real-time PCR according to the Maxima SYBR Green/SYBR qPCR mix instructions. All reactions were repeated three times, and the reaction conditions were as follows: 5 min at 95°C, followed by 40 cycles at 95°C for 10 s, 58°C for 20 s, and 72°C for 20 s. *β*-Actin was used as an internal reference to normalize target levels of TRPV1 and TNF-*α* mRNA in the endometrium. The primer sequences are shown in Table 1.

### 2.10. Statistical Analysis

SPSS 20.0 software was used for data processing and statistical analysis. The measurement data were expressed as the mean ± standard deviation (‾*x* ± *s*), and the normality and homogeneity of the variance were tested. A one-way analysis of variance was used for comparison among multiple groups. The LSD test was used when the variance of the pairwise comparison between the groups was homogeneous, and Dunnett's T3 test was used when the variance was uneven. *P* value <0.05 indicated that the difference was statistically significant.

The flowchart of the animal experiments used in this study is summarized in Figure 1.

## 3. Results

### 3.1. Effects of HYSJ-EL on the Thermal Pain Threshold in Rats with Endometriosis

As shown in Figure 2, four weeks after modeling, compared to the sham group, the thermal pain threshold of the other treatment groups was significantly decreased (*P* < 0.01). Eight weeks after modeling, there was no significant difference in the thermal pain threshold of the model group compared to before administration (*P* > 0.05). The thermal pain threshold of the HYSJ-EL group and the positive control group was higher than before administration (*P* > 0.05). After 4 weeks of modeling, compared with the normal control group, the thermal pain threshold of the three groups significantly decreased (*P* < 0.01). After 8 weeks of modeling, compared with the normal control group, the thermal pain threshold in the model group had decreased (*P* < 0.01). Compared with the model group, the thermal pain threshold of the positive control group and the enema group was significantly increased (*P* < 0.01). Compared with the positive control group, the thermal pain threshold of the HYSJ-EL group decreased (*P* < 0.01).

### 3.2. Effects of HYSJ-EL on Endometrial Histomorphology in Rats with Endometriosis

As shown in Figure 3, in the normal control group, the endometrial epithelium of the rats was intact, the columnar epithelial cells were continuously and orderly arranged, the interstitial cells were densely and orderly arranged, and the microvilli were dense. In the ectopic endometrium of the model group, columnar, flat, and cubic epithelial cells proliferated, interstitial cells proliferated intensively, and glands were visible. The ectopic endometrium of the indomethacin group and the HYSJ-EL group showed a dense and irregular arrangement of columnar epithelial cells, an uneven density of stromal cells, and glands were visible.

### 3.3. Effects of HYSJ-EL on Lesion Size in Rats with Endometriosis

There was no ectopic lesion in the sham operation group, and the lesion size was recorded as 0. As shown in Figure 4, compared with the sham operation group, the ectopic lesions in the model group were significantly increased (*P* < 0.01). Compared with the model group, ectopic lesions in the indomethacin group and HYSJ-EL group were decreased (*P* < 0.01). Compared with the indomethacin group, the lesion size in the HYSJ-EL group was not significantly different (*P* > 0.05).

### 3.4. Effects of HYSJ-EL on Masson Staining in Rats with Endometriosis

The fibers were colored in blue following Masson staining. As shown in Figure 5, a small amount of fiber staining was observed in the endometrium of rats in the normal control group, and a large number of fiber staining was observed in ectopic lesions, which were mainly distributed in the stroma. Compared with the normal control group, the fibrosis area ratio of ectopic lesions in the model group increased, and the difference was statistically significant (*P* < 0.01). Compared with the model group, the fibrosis area ratio of ectopic lesions in the indomethacin group and the HYSJ-EL group decreased, and the difference was statistically significant (*P* < 0.01). Compared with the indomethacin group, there was no significant difference in fibrosis area ratio in the HYSJ-EL group (*P* > 0.05).

### 3.5. Effects of HYSJ-EL on the Level of PGE2, IL-6, and MIP-2 in the Serum of Rats with Endometriosis

As shown in Figure 6, compared to the normal control group, the serum concentrations of PGE2, IL-6, and MIP-2 in the model group increased (*P* < 0.01). Compared to the model group, the PGE2, IL-6, and MIP-2 concentrations in the HYSJ-EL group and in the indomethacin group decreased (*P* < 0.01). Compared with the indomethacin group, the concentrations of PGE2, IL-6, and MIP-2 in the HYSJ-EL group increased (*P* < 0.01).

### 3.6. Effects of HYSJ-EL on TGF-*β* and PAI-1 Levels in the Serum of Rats with Endometriosis

As shown in Figure 7, compared to the sham operation group, the concentrations of TGF-*β* and PAI-1 in the serum of rats in the model group increased (*P* < 0.01). Compared to the model group, the concentrations of TGF-*β* and PAI-1 in the HYSJ-EL group and the positive control group decreased (*P* < 0.01). Compared with the indomethacin group, the concentrations of TGF-*β* and PAI-1 in HYSJ-EL group increased (*P* < 0.01).

### 3.7. Effects of HYSJ-EL on Endometrial Expression of TRPV1 and TNF-*α* Protein and mRNA in Rats with Endometriosis

As shown in Figure 8, compared to the eutopic endometrium of the sham operation group, the expression of TRPV1 and TNF-*α* protein and mRNA in the ectopic endometrium of the model group increased (*P* < 0.05). Compared to the model group, the expression of TRPV1 and TNF-*α* protein and mRNA in the HYSJ-EL group and in the positive control group decreased (*P* < 0.01). Compared with the indomethacin group, the expression of TRPV1 and TNF-*α* in the HYSJ-EL group increased (*P* < 0.01).

## 4. Discussion

In this study, we focused on the effects of Huayu Sanjie enema liquid on EMs model rats. TCM sustains that the basic pathogenesis of EMs is due to “blood stasis” blocking the uterus in the Chong and Ren channels, and the treatment method mainly promotes blood circulation to remove blood stasis. Modern pharmacological studies have shown that the Taohong Siwu decoction, *Sparganii Rhizoma, Rhizoma Curcumae,* and *Radix Salviae Miltiorrhizae* in Huayu Sanjie Enema Liquid exert effects of anti-inflammatory, analgesia, improving hemodynamics, and stimulating the immune response [20]. Compared to oral administration of TCM preparations, a TCM enema preparation for the treatment of pelvic pain has the advantages of directly reaching the location of the disease, easy absorption, avoiding the liver first-pass effect, and reducing gastrointestinal stimulation [21]. Previous clinical studies have shown that the Huayu Sanjie Enema Liquid can achieve good clinical effects in the treatment of EMs and can significantly improve the pain symptoms of EMs patients and improve their quality of life [22].

Currently, the mechanisms underlying pelvic pain in EMs are not fully understood. Recent studies have found that the inflammatory response, peripheral nerve sensitization, and pelvic adhesion are involved in the generation of pelvic pain in EMs. They interact with each other, directly or indirectly to stimulate nerve endings or mediate the sensitivity of nerve endings, thus inducing pain [23, 24].

In this study, we evaluated the relieving effect of Huayu Sanjie Enema Liquid on pelvic pain in rats with EMs using the thermal pain threshold test and determined the expression levels of pain-related factors PGE2 and TRPV1. PGE2 is the main pain factor and inflammatory factor of EMs [25, 26]. The elevated PGE2 in the serum and peritoneal fluid of EMs patients can cause uterine smooth muscle contraction, reduce uterine blood flow, and lead to uterine ischemia and hypoxia, accumulation of acidic metabolites, and pain [8]. Local high prostaglandin levels in EMs lesions can induce the inflammatory response, increase vascular permeability, and activate bradykinin levels, causing local hyperalgesia and pain.

TRPV1 is a channel protein closely related to peripheral sensitization of pain. Peripheral sensitization refers to an increase in the excitability of peripheral nociceptors to nociceptive stimuli. Peripheral sensitization is an important link in the establishment of pelvic pain in EMs. When inflammation occurs in the ectopic lesion of EMs, various inflammatory factors are released by the local and surrounding cells of the lesion. These inflammatory factors will initiate a series of signaling pathways, thus activating or sensitizing the relevant ion channels located on the end surface of the nociceptors, stimulating the nociceptors, and causing pain [27]. TRPV1 is a nonselective ligand-gated cation channel widely distributed in nociceptors, which is closely related to pain transmission [28]. TRPV1 plays an important role in the formation of nociceptive thermal sensation and pathological thermal hyperalgesia. Studies have found that TRPV1 is essential for thermal hyperalgesia caused by inflammation and tissue damage. The reactivity of TRPV1-knockout mice to nociceptive thermal stimulation is significantly reduced, and the thermal hyperalgesia in the inflammatory environment is significantly weakened [29, 30]. Studies have shown that the expression of TRPV1 is positively correlated with the degree of chronic pelvic pain in peritoneal lesions and sacral ligament lesions in patients with EMs, and the density of TRPV1 positive nerve fibers positively correlates with the severity of dysmenorrhea [31]. TRPV1 is regulated by a variety of inflammatory factors, which can directly or indirectly activate TRPV1, thus triggering or promoting pelvic pain in EMs. After TRPV1 is sensitized by inflammation, its activation threshold is significantly reduced, resulting in hyperalgesia and pain hypersensitivity. Studies have shown that in the presence of prostaglandins, the temperature threshold of TRPV1 activation is reduced to below 35°C, allowing TRPV1 to be activated at normal body temperature and the induction of spontaneous pain. TNF-*α* can bind to TRPV1, thus regulating the current of the voltage-gated sodium channel, inducing the continuous potential of the sensory nerve, increasing the current in the nerve fibers, and causing pain [32]. In bone cancer pain model rats, IL-6 can up-regulate the expression of the TRPV1 protein in the dorsal root ganglia through the Janus kinase (JAK)/phosphatidylinositol 3-kinase (PI3K) pathway and participate in peripheral sensitization [33]. Furthermore, in endometrial epithelial mesenchymal cells with EMs, TNF-*α* and PGE2 can stimulate the expression of TRPV1, and TRPV1 further induces the release of factors such as nitric oxide (NO) and interleukin IL-1*β* to promote the development of inflammation [34]. This study found that compared to the sham operation group, the thermal pain threshold of the model group decreased, TRPV1 and TNF-*α* protein were highly expressed in ectopic lesions, and serum expression of IL-6 and PGE2 increased. It is speculated that this process may involve TNF-*α*, PGE2, IL-6, and other inflammatory factors that upregulate and activate TRPV1, causing thermal hyperalgesia and pelvic pain observed in EMs.

The results of this study showed that when compared with the normal control group, the thermal pain threshold of the model group was decreased (*P* < 0.01), the serum PGE2 concentration was increased (*P* < 0.01), and the expression of TRPV1 protein and mRNA in ectopic endometrium was increased (*P* < 0.01) after 4 weeks of modeling, which indicated that there was pelvic pain in the EMs model rats, and the expression levels of PGE2 and TRPV1 were increased. Compared with the model group, the heat pain threshold of the indomethacin group and the HYSJ-EL group increased (*P* < 0.01), the serum PGE2 concentration decreased (*P* < 0.05), and the protein and mRNA expression of TRPV1 in ectopic endometrium decreased (*P* < 0.05), indicating that Huayu Sanjie enema liquid could relieve the pain of the EMs model rats and influence the expression of PGE2 and TRPV1.

EMs has long been considered an aseptic inflammatory disease [35]. Its occurrence and development and the production of pelvic pain are related to the mediation of many inflammatory factors [36, 37]. In this study, we measured the expression levels of PGE2, IL-6, TNF-*α*, and MIP-2 to evaluate the effects of Huayu Sanjie enema on inflammation. IL-6 and TNF-*α* are important cytokines involved in various inflammatory and immune responses in the human body [38]. Studies have shown that IL-6 and TNF-*α* can promote the occurrence and development of EMs and are expressed in patients with EMs [7, 9]. Enhanced levels can further induce the release of inflammatory factors and participate in immune damage [39]. At the same time, TNF-*α* promotes the formation of new blood vessels and can stimulate the proliferation of endometrial stromal cells and promote the adhesion of endometrial cells, increase the adhesion of endometrial stroma with mesothelial cells and surrounding tissues, which are all factors contributing to the occurrence and development of EMs [40]. Macrophage inflammatory protein-2 (MIP-2) is a chemokine widely involved in immune inflammatory activity and angiogenesis. Studies have found that the expression of IL-6, TNF-*α*, and MIP-2 in patients with EMs increased, thus inducing the inflammatory response and promoting the implantation and growth of the ectopic endometrium [6, 41]. This study found that compared to the sham operation group, the expression of IL-6, PGE2, and MIP-2 in serum and TNF-*α* protein in ectopic lesions of rats in the model group was higher, suggesting that the EMs rat model exerted an inflammatory response, which was related to pain in rats.

Most patients with EMs present different degrees of pelvic adhesions. Inflammatory pathological processes can lead to pelvic fibrosis and adhesions. The fibrous fascicles formed by the adhesions will stretch or twist tissues and organs. Nerve fibers in stretched tissues and organs will produce impulses to the central nervous system, which produce pain in their corresponding cortex area. TGF-*β* can promote fibroblast proliferation, collagen deposition, and fibrin formation, increase extracellular matrix collagen synthesis, and reduce degradation which leads to pelvic fibrosis and adhesions and promotes the development of EMs [42]. PAI-1 is an antifibrinolytic factor that can antagonize plasminogen-induced extracellular matrix degradation, promote fibrin formation, and promote the appearance of adhesions [43]. This study found that compared to the blank control group, the expression levels of PAI-1 and TGF-*β* in the serum of the model group increased, suggesting that there may be pelvic adhesions in rats models of EMs, and PAI-1 and TGF-*β* are related to pain in rats.

In addition, this study evaluated the analgesic effects of Huayu Sanjie Enema Liquid on EMs rats and its effects on inflammation, peripheral sensitization, and pelvic adhesions. The results showed that compared to the model group, the thermal pain threshold of the HYSJ-EL group and the indomethacin positive control group significantly increased, serum levels of PGE2, IL-6, MIP-2, PAI-1, and TGF-*β* decreased, and TRPV1 and TNF-*α* protein expression in tissues of ectopic lesion significantly decreased. Compared with the indomethacin group, the HYSJ-EL group had similar efficacy in improving lesion size and reducing fibrosis. Although the effect of the HYSJ-EL group in reducing inflammatory response and pain was not as effective as that of the indomethacin group, considering the common adverse reactions of indomethacin on the gastrointestinal tract [44, 45], TCM enema may have good application prospects in the treatment of EMs.

## 5. Conclusions

In summary, Huayu Sanjie enema can play a role in the therapeutic effect on EMs by inhibiting the lesion size, fibrosis, and pelvic pain of EMs model rats. The mechanism may be that Huayu Sanjie Enema Liquid inhibits the expression of PGE2, IL-6, MIP-2, TNF-*α*, PAI-1, TGF-*β*, and TRPV1, thereby inhibiting its mediated inflammatory response, peripheral sensitization, and pelvic adhesion, thus alleviating the pelvic pain in rats with EMs.

## Figures and Tables

**Figure 1:** Flowchart of the animal experiments.

**Figure 2:** The thermal pain threshold at 4 and 8 weeks.  ^*∗∗*^*P* < 0.01, compared to the normal control group.  ^##^*P* < 0.01, compared to the model group.  ^∧∧^*P* < 0.01, compared to the indomethacin group.

**Figure 3:** The morphology of the endometrial tissue of each group. Black arrows show epithelial cells; blue arrows show glands.

**Figure 4:** The size of the lesions in each group. In the bar charts,  ^*∗∗*^*P* < 0.01, compared to the normal control group.  ^##^*P* < 0.01, compared to the model group.

**Figure 5:** The lesion fibrosis in each group. In the bar charts,  ^*∗∗*^*P* < 0.01, compared to the normal control group.  ^##^*P* < 0.01, compared to the model group.

**Figure 6:** Serum levels of PGE2, IL-6 and MIP-2. In the bar charts,  ^*∗∗*^*P* < 0.01, compared to the normal control group.  ^##^*P* < 0.01, compared to the model group.  ^∧∧^*P* < 0.0, compared to the indomethacin group.

**Figure 7:** The serum levels of TGF-*β* and PAI-1. In the bar charts,  ^*∗∗*^*P* < 0.01, compared to the normal control group.  ^##^*P* < 0.01, compared to the model group.  ^∧∧^*P* < 0.0, compared to the indomethacin group.

**Figure 8:** TRPV1 and TNF-*α* protein and mRNA expression in the endometriotic tissues. In the bar charts,  ^*∗*^*P* < 0.05, compared to the normal control group.  ^*∗∗*^*P* < 0.01, compared to the normal control group.  ^##^*P* < 0.01, compared to the model group.  ^∧∧^*P* < 0.01, compared to the indomethacin group.

**Table 1:** Primer sequence.

Name	Primer sequence
*β*-Actin	F: CTATCGGAATGAGCGGTTC
	R: CTTAGGAGTTGGGGGTGGCT

TNF-*α*	F: ACCACGCTCTTCTGTCTACTG
	R: CTTGGTGGTTTGCTACGAC

TRPV1	F: CCAACGCAAGGAGTATGTGG
	R: GACGAACATAAACCGGCACA

## Data Availability

The data used to support the findings of this study are available from the corresponding author upon request.
